This article has been retracted.

# Feasibility Study on the Integration of Innovation and Entrepreneurship Education and Occupational Therapy Training Mode for College Students Based on Big Data

**DOI:** 10.1155/2022/3911326

**Published:** 2022-05-09

**Authors:** Yan Yang, Juan Xie

**Affiliations:** ^1^Department of Innovation and Entrepreneurship, Hunan Institute of Technology, Hengyang, Hunan 421002, China; ^2^Department of Computer Science and Engineering, Hunan Institute of Technology, Hengyang, Hunan 421002, China

## Abstract

With the development of information technology, the status of the traditional teaching method combining chalk and blackboard is declining. People need a novel teaching method to reform traditional education, so the hybrid teaching mode combining the advantages of both is produced and has become a major research hotspot in the field of education technology at present. Further accelerating the reform of innovation and entrepreneurship teaching in higher education institutions and improving students' innovation and entrepreneurial ability based on big data technology are the fundamental measures to do a good job in managing college students' entrepreneurship and employment. Therefore, the reform of dual-innovation education in colleges and universities has become a research hotspot in recent years. How to combine the two aforementioned research hotspots in order to improve college students' dual-innovation ability is a key issue that needs to be solved urgently. College students' innovation and entrepreneurship practice is in full swing in colleges and universities, but the success rate of college students' entrepreneurship is not high. In order to promote the development of college students' entrepreneurial practice, colleges and universities can give them the necessary help. Integrating the content of “dual innovation” education with big data technology into the ideological and political education of college students can not only improve the ideological and political quality and moral and psychological quality of college students but also convey the relevant legal policies of innovation and entrepreneurship to college students. Today's society has entered the Internet era, the resource of information technology, and the rapid development of the Internet which provides good technical support and rich content choices for the innovation of ideological and political education of college students in the context of “dual innovation,” but it also poses new challenges for the ideological and political education of college students. By studying the exercise data of groups at all levels in the campus, we analyze and compare the overall exercise situation of each type of group and explore and study the overall exercise situation of various classes, grades, schools, etc., to understand the physical activity. We can build a group of ideological and political education teachers with innovative and entrepreneurial literacy based on big data analysis. Only in this way can the ideological and political education of college students really give some help to the practice of innovation and entrepreneurship of college students and stimulate the potential of innovation and entrepreneurship of college students from a deeper level.

## 1. Introduction

Since the late 1980s, with the rapid development of information technology, E-learning has become popular around the world. People want to use E-learning to reform the traditional classroom teaching [1]. By the end of the twentieth century, the shortcomings of E-learning caused people to reflect on the process of using E-learning and blended learning emerged for the first time in corporate training as an alternative to E-learning [2]. With the continuous exploration of this new learning method, the integration of online learning and face-to-face teaching was gradually realized. Since then, blended learning has been commonly used in the field of education and has gained surprising training utility [3]. In recent years, the attention of foreign scholars to blended learning has caused domestic scholars to discuss and conduct in-depth research on blended learning. At this stage, in the new historical context, blended learning manifests new meanings [4]. How to use educational technology to improve teaching quality and comprehensively improve the quality of talent cultivation has become an urgent need in China's educational practice. First of all, innovation education is the foundation in entrepreneurship education, providing more theoretical help for entrepreneurship education, so that the level of entrepreneurship education can be further improved [5]. From another perspective, entrepreneurship education can also be regarded as the carrier and expression of innovation education, all of which is intended to be operable and practical. Unlike other forms of education, innovation and entrepreneurship education is more focused on the quality of education and more precise for the cultivation of talents [6–9]. Innovative entrepreneurship education harmonizes talents with national economic development and social needs. By sorting out the above concepts of innovation and entrepreneurship education, the innovation and entrepreneurship education to be studied in this paper specifically refers to the improvement of students' innovation and entrepreneurial ability through various educational teaching [10].

Innovation is the first driving force leading development, entrepreneurship is an important driving force for national economic development and social value creation, and innovation and entrepreneurship activities assume the role of a bridge and link to transform science and technology into productivity [11]. The process of worldwide economic integration is accelerating, the scientific and technological revolution and industrial changes are taking place, and the international economic landscape is also undergoing significant changes. Facing the changes of macro environment, each country gradually realizes that it is necessary to promote the manufacturing industry from factor and investment driven to innovation driven and add new vitality to the manufacturing industry with science and technology innovation [12]. Innovation has become an important strategy for international competition and an important driving force to lead the development of each country [13]. In such a background, China, as a large manufacturing country, is facing the problem of “all but not fine, big but not strong,” and the demographic dividend is gradually disappearing, leading to a gradual slowdown of China's economic development. Innovation-driven development strategy is an important strategy to lead China's economy to develop in the direction of high speed and high quality, and it is necessary to stimulate the huge potential of innovation in a wider scope, wider space, and deeper field and promote the construction of an innovative country and a world scientific and technological power [14]. Rich theory of dual innovation education provides theoretical support to improve the effectiveness of dual innovation education in colleges and universities [15]. Entrepreneurship rate is usually taken as an important index to measure the effectiveness of innovation and entrepreneurship education in colleges and universities [16]. However, this study believes that the entrepreneurship rate of college students, as a single data indicator, can only reflect the one-sided situation of innovation and entrepreneurship education in colleges and universities, not the comprehensive results [17–19]. From the perspective of the ultimate purpose of dual innovation education, it is not to promote students' entrepreneurship and enhance the employment rate, but more importantly to promote the development of students' comprehensive quality in all aspects [20]. Based on this, this study selects two indicators, innovation spirit and entrepreneurial ability, to examine the impact of dual-innovation education on students' development, and then analyzes effective countermeasures and suggestions that are beneficial to students' development [21].

This study is relevant to current affairs and can provide some reference for the national education sector. According to the current national policies, the state is exploring the way of deep integration of information technology and education, trying to build a new model of talent cultivation under the condition of “Internet+,” and encouraging universities to form a “dual creation pattern combining online and offline,” but no solution has been found yet. This study provides a preliminary exploration of the solution to this problem and provides some ideas for the relevant departments. This study meets the needs of real life. In reality, we can see the phenomenon of failure of college students' entrepreneurship everywhere. The fundamental way to improve the employment rate of college students is to improve their ability of dual innovation. College students usually live in universities, so the responsibility of improving college students' dual-innovation ability lies in colleges and universities to promote dual-innovation education reform deeply. Up to now, several years have passed since the implementation of double-creative education in colleges and universities, but how effective is it? Has it effectively improved the students' ability of dual innovation? These are not yet known. This study can take this opportunity to investigate the development of dual-innovation education in some regions and provide reference for the relevant national departments. It can be said that this study is of great practical significance for the country to speed up the implementation of innovation-driven development strategy, accelerate the reform and development of higher education, and promote high-quality entrepreneurship and employment of college graduates.

## 2. Methods

### 2.1. Design

Most foreign academics agree that entrepreneurship education is a product of modern social development and is needed and driven by entrepreneurial economic development and that entrepreneurial talents are needed by modern society. Therefore, the concept of entrepreneurship education should better cultivate entrepreneurial consciousness, entrepreneurial spirit, and entrepreneurial ability, to improve the overall quality of entrepreneurs. Peter F. Drucker, the father of modern management and a professor at Claremont Graduate University, once said, “Entrepreneurship is not a magical inaccessible thing, it is not an innate ability. Entrepreneurship is a method of learning and training, and like any knowledge, it can be mastered through learning.” Many scholars agree with this statement. For example, scholar Ronstadt (Ronstadt) believes that entrepreneurship education is a forward-looking educational model through which more people with entrepreneurial talent can be developed and that entrepreneurship education can actually enhance not only entrepreneurial opportunities but also more potential jobs. Professor Gibb even argues that virtually every student has an entrepreneurial soul running through their own blood and growing an entrepreneurial vein, and that entrepreneurship education can solidify these students' talents and put them into practice. But entrepreneurs, like some artists, must have a good foundation to become a good artist, and a good entrepreneurship education is the foundation of those foundations.

### 2.2. Participants

The earliest research on entrepreneurship education was conducted in the U.S., and the research on innovation education for college students in the U.S. is still far ahead of other countries. In 1945, Harvard University proposed in its book “General Education in a Free Society” that schools should know how to develop students' innovative thinking ability in their daily learning process. At present, by searching the special literature, we find that the scholars' research on innovation education mainly discusses the innovation education of college students from two aspects. One is to analyze the innovation education of college students from theory, and the other is to argue the innovation education of college students in practice. For example, the Massachusetts Institute of Technology (MIT) in the United States, in the process of cultivating students' innovation education, uses a combination of learning inside and outside the classroom to purposefully plan students' research work (UROP for short), and students can choose a topic to research according to their own interests and invite teachers to join them as soon as they enroll. In addition, students can also choose to work independently on their project activities and choose different ways to collaborate according to their needs. These books and journals will not only provide students with more platforms for development, but will also truly motivate American colleges and universities to enhance the development of innovative education. For example, Shana Daly et al. argue in “Innovative Educational Perspectives on Interdisciplinary Studies for Undergraduates” that the “innovation process” is the creative use of new modes of thinking and new learning experiences by students in the learning process. Teachers focus on the use of innovative factors in the teaching process, which is conducive to broadening teaching channels, updating teaching concepts, and truly cultivating students' innovative thinking and abilities. In addition, there are some scholars with different views.

There are many factors that influence whether an individual will start a business or not, and a few representative points are pointed out for analysis and research: social environment in the context of the times, education level, life experience, personal temperament, personality, and other related factors. Among them, people with extroverted personality traits have the highest tendency to start their own business.

### 2.3. Measures

In the field of “double-creation” education, ideological and political education activities can use both positive and negative entrepreneurial models or exemplars to propagate, promote, and reflect, so as to achieve the role of demonstration, guidance, and education, which is the main way of typical education method in ideological and political education. This is the main way of typical education in ideological and political education. For the “double creation” activities, ideological and political education can be carried out through the successful entrepreneurial typical, so that college students can study and learn from the thoughts and behaviors of the typical or role model and then internalize them. In addition, failed entrepreneurial cases can also be used as negative teaching materials to guide and educate college students, through which college students are warned not to blindly follow and imitate, so that they can learn lessons from the negative examples. College students often have a strong imitation mentality, which comes from their inner needs and the influence of social herd mentality. Therefore, the ideological and political education work should correctly perceive and accurately grasp the psychological needs of college students under the perspective of “double creation” education and guide them to actively learn from various typical examples. Through learning from positive examples, students should learn their successful experiences and praiseworthy spiritual qualities of innovation and entrepreneurship; at the same time, they should learn from the failed cases and improve themselves. The use of typical education method has the following characteristics.

Visualization. In the field of “double-innovation” education, one of the purposes of model education method is to establish and publicize typical entrepreneurship, that is, to visualize the abstract theoretical content and spiritual essence through the successful or unsuccessful cases of real entrepreneurs. It makes college students have a clear understanding and resonate with them. This exemplary nature mainly refers to the experience, methods, spirit, and qualities in the typical entrepreneurship which are positive and can be learned and studied. In the process of entrepreneurship, college students should study and learn from the entrepreneurial ideas and spirit of the typical entrepreneur. Infectious. Entrepreneurial models tend to be more persuasive and attractive, and positive entrepreneurial models are even more so. They can guide and educate college students with their personal experiences and lessons learned in the process of entrepreneurship, to promote their worship and admiration and further trigger their motivation to imitate and promote the formation of the situation of catching up and learning.

## 3. Bi-Innovation and Occupational Therapy Integration

### 3.1. Demographic Variability Test

It has been shown that students' innovativeness and entrepreneurship are influenced by demographic variables. In this study, the six variables of gender, grade level, type of major, and type of institution, whether there are close relatives to start a business, and home location were selected, and the significant difference test revealed that students' innovative spirit and entrepreneurial ability were significantly different on the four variables of gender, grade level, type of school, and close relatives to start a business, while the two variables of professional type and home place on innovative spirit and entrepreneurial ability were independent samples *t*-test analysis; the results are shown in Table 1. From Table 1, it can be seen that the two variables of innovation and entrepreneurial ability differ significantly by gender among college students, specifically, male students have significantly higher innovation and entrepreneurial ability than female students. There were no significant differences in either ground.

The results of the one-way ANOVA for the two variables of innovation and entrepreneurial ability at the student's grade level are shown in Table 2. From Table 2, it can be seen that the variables of innovative spirit and entrepreneurial ability are significantly different at each student's grade level. In general, innovation and entrepreneurial ability were higher in the upper grades than in the lower grades. Specifically, in terms of innovation spirit, senior > sophomore > freshman, junior > freshman, and junior > freshman, while there was no significant difference between juniors and seniors. In terms of entrepreneurial ability, sophomore, junior, and senior years were all higher than freshman year, while there was no significant difference between the senior years.

The results of the independent sample *t*-test analysis of the two variables, innovation and entrepreneurial ability, on the type of institution are shown in Table 3. From Table 3, it can be seen that the variables of innovation and entrepreneurial ability differ significantly in the type of college, which indicates that the different types of institutions have different effects on students' innovation and entrepreneurial ability. Specifically, students from key institutions have significantly higher innovation spirit and entrepreneurial ability than students from ordinary institutions.

### 3.2. Feasibility Analysis of Occupational Therapy Training Model

In this study, dual-innovation education is divided into three forms: theoretical courses, practical activities, and professional courses integrated into dual-innovation education. Since professional courses integrated into dual-innovation education essentially refer to professional course education, which is mandatory for students to participate, they are not considered here. Theoretical courses (e.g., elective courses) and practical activities (e.g., creative projects), on the other hand, always adhere to the principle of students' voluntary participation, so the degree of participation of different students in these two forms of dual-innovation education is bound to be different. The effectiveness of dual-innovation education can be reflected from the perspective of “quantity.” Theoretical courses include compulsory courses, elective courses, and related lectures. Except for compulsory courses, other types of courses always adhere to the principle of students' voluntary participation, so there are certain differences in the degree of participation of different students in theoretical courses. A one-way ANOVA was conducted on the variables of innovation and entrepreneurial ability for students with different levels of participation in theory courses, and the results are shown in Figure 1: the mean values of innovation for students with no participation, occasional participation, and frequent participation were 2.9448, 3.3584, and 3.6028, respectively, and the mean values of entrepreneurial ability were 2.7401, 3.1847, and 3.4112, respectively, with a gradual increasing trend, and the *F*-value of innovation was 15.006, *p* < 0.01, and the *F*-value of entrepreneurial ability was 16.655, *p* < 0.01, all of which were significantly different. After post hoc comparison (LSD), students' innovative spirit and entrepreneurial ability were related to the degree of participation in the dual-innovation theory course, specifically, frequently > occasionally involved > not involved, i.e., students who were frequently involved had higher innovative spirit and entrepreneurial ability than those who were occasionally involved and much higher than those who were not.

Practical activities, including entrepreneurship projects, entrepreneurship training, and entrepreneurship plan competition, also consistently adhere to the principle of voluntary student participation, so there will be some differences in the degree of participation of different students in practical activities. The results of the one-way ANOVA on the variables of innovation spirit and entrepreneurial ability among students with different levels of participation in practical activities are shown in Figure 2; the mean values of innovation spirit for students who did not participate, occasionally participated, and frequently participated were 2.8531, 3.3088, and 3.7411, respectively, and the mean values of entrepreneurial ability were 2.6621, 3.2272, and 3.4467, respectively, with a gradual increasing trend. The *F*-value for innovative spirit was 28.783, *p* < 0.01, and the *F*-value for entrepreneurial ability was 21.218, *p* < 0.01, both of which were significantly different. After post hoc comparison (LSD), students' innovative spirit and entrepreneurial ability were related to the degree of participation in courses and activities related to dual-innovation education, specifically, often > occasionally involved > not involved, i.e., students who were often involved had higher innovative spirit and entrepreneurial ability than those who were occasionally involved and much higher than those who were not. When students feel better about a certain type of dual-innovation education, it means that the better the quality of this type of dual-innovation education is, the greater the impact on students, and the more conducive to the development of students' innovation and entrepreneurship.

Therefore, to investigate the relationship between students' feelings about different forms of dual-innovation education and their innovation and entrepreneurial ability, we can reflect the effectiveness of dual-innovation education from the perspective of “quality.” An independent sample *t*-test was conducted on the variables of innovation and entrepreneurial ability for students with different perceptions of the harvest of the theoretical courses: the mean values of innovation and entrepreneurial ability for students with low perceptions of the harvest were 2.9684 and 2.8617, while the mean values of innovation and entrepreneurial ability for students with high perceptions of the harvest were 3.4495 and 3.3728, and *p* was less than 0.01, which were significantly different. It indicates that the improvement of students' innovative spirit and entrepreneurial ability are related to the degree of gain in the theoretical course, specifically, students with high sense of gain in the theoretical course have higher innovative spirit and entrepreneurial ability than students with low sense of gain.

### 3.3. Analysis of Variability in the Degree of Integration

The results of the independent sample *t*-test on the variables of innovative spirit and entrepreneurial ability for students with different perceptions of the degree of integration between dual-innovation education and professional education are shown in Figure 3; the mean value of innovative spirit for students with low perceptions of integration is 2.9946, and the mean value of entrepreneurial ability is 2.9075, while the mean value of innovative spirit for students with high perceptions of integration is 3.4619 and the mean value of entrepreneurial ability is 3.3755. The mean value of innovative spirit and entrepreneurial ability of the students who thought the combination of both was high was 3.4619, and the mean value of entrepreneurial ability was 3.3755. The results indicate that students' innovative spirit and entrepreneurial ability are related to the degree of integration of dual-innovation education and professional education in the perceived degree of integration, specifically, students with high perception of integration of dual-innovation education and professional education have higher innovative spirit and entrepreneurial ability than students with low perception. The reasons for this may be due to, first, the fact that this form of dual-innovation education generally focuses on imparting a systematic knowledge structure and generally uses a didactic approach, which is not conducive to student initiative.

In order to reliably determine the quality variables of different forms of dual-innovation education, this study uses students' feelings about different forms of dual-innovation education to indicate the high and low quality of dual-innovation education, i.e., the better students' feelings about a certain form of dual-innovation, the higher the quality of that form of dual-innovation education.

From the degree of students' acceptance of dual-innovation education and the evaluation of students' perceptions of dual-innovation education, it can be concluded that different forms of dual-innovation education can effectively promote the development of students' innovation and entrepreneurship. In order to further investigate the differences in the degree of influence of three different forms of dual-innovation education on students' development, namely, theoretical courses, practical activities, and professional courses integrated with dual-innovation education. This study establishes a regression model between students' perceptions of different forms of dual-innovation education and students' innovation and entrepreneurial abilities. Based on this, this study establishes regression models for students' feelings about the three types of dual-innovation education with innovation spirit and entrepreneurial ability, respectively, and then analyzes the size of the influence of different types of dual-innovation education on students' development according to the regression coefficients. The different feelings of students towards theoretical courses, practical activities, and professional courses integrated with dual-innovation education are regressed with the innovation spirit of college students. The *R*-squared of the regression model after putting the three forms of dual-innovation education into it becomes 0.357, and the significance level is still 0.000. It indicates that the three forms of dual-innovation education can explain 35.7% of the variance of students' innovative spirit. The regression coefficient of practical activity education and innovative spirit is 0.520 and 0.000, which indicates that practical activity can significantly and positively predict innovative spirit; similarly, it indicates that theoretical courses and professional courses integrated into dual-innovation education can significantly and positively predict innovative spirit; based on the magnitude of the regression coefficient, it can be seen that practical activity has the greatest impact on innovative spirit, followed by theoretical courses, and integrated into professional education The impact of dual-innovation education is the smallest.

## 4. Regression Analysis of Dual Innovation Education on Entrepreneurship

A regression analysis was done to correlate students' different perceptions of theoretical courses, practical activities, and professional courses integrated into dual-innovation education with college students' entrepreneurial ability. The *R*-squared of the regression model after putting the three forms of dual-innovation education into the regression model still has a significance level of 0.0001, indicating that the three forms of dual-innovation education can explain 33.2% of the variance in students' entrepreneurial ability. The regression coefficient of 0.661 with a significance level of 0.000 indicates that practical activities can significantly and positively predict entrepreneurial ability; similarly, it shows that theoretical courses and professional courses that incorporate dual-innovation education can also significantly and positively predict entrepreneurial ability. The logic lies in the fact that students are the most direct participants and beneficiaries of dual-innovation education, and their feelings about different forms of dual-innovation education can directly reflect the quality of different forms of dual-innovation education. Based on the magnitude of the regression coefficients, it can be seen that practical activities have the greatest effect on entrepreneurial competencies, followed by theoretical courses, and professional courses integrated into dual-innovation education have the least effect on them, as shown in Figure 4. From the output, the regression model is *Y* = 1.577 + 0.661 satisfaction with practical activities +0.368 sense of gain from theoretical courses +0.215 evaluation of professional courses integrated into dual-innovation education (*Y* is entrepreneurial competency).

There is a close relationship between school education, which plays a leading role in the physical and mental development of students. Before students enter college, especially at the high school level, they receive exam-oriented education that targets grades. Test-based education is centered on teachers' teaching materials, with a single form of teaching, usually using the lecture method, focusing on the learning of knowledge, neglecting students' initiative and potential, which is not conducive to the development of students' independent learning ability; the standardized test evaluation system stifles students' personality and creative development; in addition, school teachers prefer children who have good academic performance and do not get into trouble and these large and small factors in school. All these factors in schools, big and small, to some extent erase students' creativity and make them lack the awareness and courage to innovate. This is related to students' living environment and peer pressure: students live in similar closed peer groups for a long period of time, and during adolescence, students' own outlook on life and the world is immature and easily shaken and herd mentality arises. In situations of peer pressure and social group interaction, students are often more likely to abandon certain ideas, thoughts, or behaviors they hold and act in line with the majority in order to better integrate into the environment, thus resulting in a lack of courage to innovate. This is a reflection of the lack of educational synergy in the development of student innovation. The cultivation of students' innovative spirit requires long-term efforts from schools to create an innovative campus atmosphere, parents and teachers to protect students' curiosity, and society to accommodate diversity of personalities.

From Figure 5, it can be seen that the mean score of students' innovative spirit is 3.302 with a standard deviation of 0.481. From the mean value, the overall development of the current university students' innovative spirit is at an intermediate level. In terms of each dimension, all four dimensions are at a medium level, and there is less variability in the levels of different students, with the highest mean value of reflectiveness (*M* = 3.446, SD = 0.540) and the lowest mean value of criticality (*M* = 3.160, SD = 0.481). The mean score of current students' entrepreneurial competencies was 3.112, indicating that students' entrepreneurial competencies are at an upper-middle level. In terms of the dimensions, students scored the lowest in the ability to explore opportunities at a low level (*M* = 2.821, SD = 0.873) and the remaining five dimensions were at a medium level, with the highest being the ability to make strategic decisions (*M* = 3.264, SD = 0.749). It has been shown that students' innovation and entrepreneurship can be influenced by demographic variables. In this study, the six variables of gender, grade level, type of major, type of institution, presence of close family members in entrepreneurship, and home location were selected, and the significance of differences test revealed that there were significant differences in students' innovative spirit and entrepreneurial ability on the four variables of gender, grade level, type of school, and close family members in entrepreneurship, while there were no significant differences on the type of major and home location. Therefore, theoretical course teaching is the foundation of students' long-term development, and the more solid the foundation, the more long-term the students' development. Therefore, in the process of promoting the overall development of students' innovative spirit and entrepreneurial ability, we must focus on combining theoretical courses with practical activities, so that students can creatively solve problems and improve their practical ability on the basis of mastering a large amount of scientific and cultural knowledge.

In contrast, although theoretical courses can also promote students' development, their impact is not as strong as that of practical activities. Secondly, the lag of educational effectiveness is especially evident in theoretical teaching. “It takes ten years to grow a tree, but a hundred years to grow a man”, which reflects the long-term and continuous nature of education work and also the lagging nature of education effectiveness. Students do not propose changes immediately after receiving education, but need some time to understand, digest, absorb, apply, and finally, internalize into their own knowledge reserves or gradually manifest in their behavior. Theory teaching is different from skill training or practical activities, it has more subtle influence on students through imparting knowledge, increasing insight, and broadening horizons. This impact is far-reaching and lasting but not significant in the short term.

However, the author believes that universities should not ignore the importance of theoretical course education. Because, theoretical course education has a fundamental role in promoting the long-term development of students. Scientific literacy is the basis for the development of innovative spirit and entrepreneurial ability, and dual-innovation education in the form of theoretical courses is the important way to improve students' scientific literacy, develop their intelligence, stimulate their innovative spirit, and improve their entrepreneurial ability. If there is a lack of broad scientific and cultural theoretical knowledge, students cannot acquire a comprehensive understanding and knowledge of a certain field, and it is difficult to break through the limitations of the original cognition and make a breakthrough and innovation.

## 5. Conclusion

Based on the thinking related to big data to analyze and study a large amount of exercise information. In this paper, we monitor users' physical activity through wearable smart terminals, collect physical activity data, and quantify the physical activity by combining the corresponding data filtering. In this paper, we monitor users' physical activity through wearable smart terminals, collect physical activity data, and quantify the physical activity by combining the corresponding data filtering. After a brief introduction of the theory related to big data, we study the analysis method of sports. After a brief introduction of the theory related to big data, we study the analysis method of sports information based on big data from the perspective of sports individuals and sports groups, respectively, with respect to the characteristics of sports. Through the study of individual sports data, we can evaluate the sports situation of each student in a single day, and in addition, we can evaluate the sports trend of an individual based on the continuous physical activity performance of an individual, so that we can evaluate the sports trend of an individual based on the continuous physical activity performance of an individual, so that we can evaluate and guide the sports situation of an individual more accurately, and to a certain extent, we can also increase the supervision of students'. On the other hand, by studying the exercise data of groups at all levels in the campus, we analyze and compare the overall exercise situation of each type of group and explore and study the overall exercise situation of various classes, grades, schools, etc., to understand the physical activity.

In the future, the ideological and political education of college students really give some help to the practice of innovation and entrepreneurship of college students and stimulate the potential of innovation and entrepreneurship of college students from a deeper level.

## Figures and Tables

**Figure 1:** One-way ANOVA of innovation and entrepreneurship in different levels of participation in theoretical courses.

**Figure 2:** One-way analysis of variance of innovation and entrepreneurship on different levels of participation in practical activities.

**Figure 3:** Analysis of the variability of innovation and entrepreneurship at different levels of integration.

**Figure 4:** Regression coefficients of different forms of dual-innovation education and entrepreneurship.

**Figure 5:** Descriptive analysis of entrepreneurial competencies in general and in each dimension.

**Table 1:** Differences in innovation and entrepreneurship by gender type.

	Gender	Number of individuals	Average value	Standard deviation (SD)	*T*-value	*p* value
Spirit of innovation	Male	152	3.69	0.69	2.69^∗∗^	0.006
	Female	369	3.25	0.42		
Entrepreneurship	Male	135	3.26	0.75	2.51^∗∗^	0.012
	Female	326	3.21	0.66		

SD: standard deviation.

**Table 2:** Differences in innovation and entrepreneurship by grade type.

	Grade	Number of individuals	Average value	Standard deviation (SD)	*T*-value	*p* value
Spirit of innovation	First year	181	3.69	0.58	2.69^∗∗^	0.006
	Second year	196	3.25	0.36		
	Third year	69	3.25	0.26		
	Fourth year	95	3.69	0.29		
Entrepreneurship	First year	135	3.26	0.59	2.51^∗∗^	0.012
	Second year	159	3.21	0.67		
	Third year	69	3.58	0.63		
	Fourth year	96	3.49	0.67		

SD: standard deviation.

**Table 3:** Differences in innovative spirit and entrepreneurial ability by grade level type.

	Grade	Number of individuals	Average value	Standard deviation (SD)	*T*-value	*p* value
Spirit of innovation	First year	181	3.69	0.58	2.69^∗∗^	0.006
	Second year	196	3.25	0.36		
Entrepreneurship	First year	135	3.26	0.59	2.51^∗∗^	0.012
	Second year	159	3.21	0.67		

SD: standard deviation.

## Data Availability

The data used to support the findings of this study are available from the corresponding author upon request.

## References

[1] Kakouris A., Liargovas P. (2021). On the about/for/through framework of entrepreneurship education: a critical analysis. *Entrepreneurship Education and Pedagogy*.

[2] Cavallini F., Carpitelli A., Corsano P., Cihon T. M. (2019). Entrepreneurship education: the case of the ABA master at the University of Studies of Parma. *Journal of entrepreneurship education*.

[3] González-López M. J., Pérez-López M. C., Rodríguez-Ariza L. (2019). Clearing the hurdles in the entrepreneurial race: the role of resilience in entrepreneurship education. *Academy of Management Learning & Education*.

[4] Ramírez-Montoya M. S., Andrade-Vargas L., Rivera-Rogel D., Portuguez-Castro M. (2021). Trends for the future of education programs for professional development. *Sustainability*.

[5] Frederiksen S. H., Berglund K. (2020). Identity work in entrepreneurship education: activating, scripting and resisting the entrepreneurial self. *International Small Business Journal*.

[6] Turner T., Gianiodis P. (2018). Entrepreneurship unleashed: understanding entrepreneurial education outside of the business school. *Journal of Small Business Management*.

[7] Bazan C., Shaikh A., Frederick S. (2019). Effect of memorial university's environment & support system in shaping entrepreneurial intention of students. *Journal of Entrepreneurship Education*.

[8] Thomas E., Pugh R. (2020). From 'entrepreneurial' to 'engaged' universities: social innovation for regional development in the global south. *Regional Studies*.

[9] Brentnall C., Rodríguez I. D., Culkin N. (2018). The contribution of realist evaluation to critical analysis of the effectiveness of entrepreneurship education competitions. *Industry and Higher Education*.

[10] Meng Q., Hou B., Ni J., Xiong M., Shan C. (2019). Research on the practical teaching of mechanical drawing based on the whole-process combination. *2018 International Workshop on Education Reform and Social Sciences (ERSS 2018)*.

[11] Cunningham J. A., Lehmann E. E., Menter M., Seitz N. (2019). The impact of university focused technology transfer policies on regional innovation and entrepreneurship. *The Journal of Technology Transfer*.

[12] Seidel V. P., Marion T. J., Fixson S. K. (2020). Innovating how to learn design thinking, making, and innovation: incorporating multiple modes in teaching the innovation process. *INFORMS Transactions on Education*.

[13] Clauss T., Moussa A., Kesting T. (2018). Entrepreneurial university: a stakeholder-based conceptualisation of the current state and an agenda for future research. *International Journal of Technology Management*.

[14] Secundo G., De Carlo E., Madaro A., Maruccio G., Signore F., Ingusci E. (2019). The impact of career insight in the relation with social networks and career self-management: preliminary evidences from the Italian contamination lab. *Sustainability*.

[15] Peng M. Y. P., Chen C. C. (2019). The effect of instructor's learning modes on deep approach to student learning and learning outcomes. *Educational Sciences: Theory & Practice*.

[16] Yiying X. (2021). Strengthening practice teaching and improving college students' innovative practice. *Advances in Vocational and Technical Education*.

[17] Olelewe C. J., Agomuo E. E., Obichukwu P. U. (2019). Effects of B-learning and F2F on college students' engagement and retention in QBASIC programming. *Education and Information Technologies*.

[18] Wang J., Tan Y. (2020). Social factory as prosaic state space: redefining labour in China's mass innovation/mass entrepreneurship campaign. *Environment and Planning A: Economy and Space*.

[19] Okori O. A., Ebere O. J. (2019). Science and mathematics education as tools for developing entrepreneurship skills among secondary school students in cross river state, Nigeria. *Global Journal of Educational Research*.

[20] Wagner M., Schaltegger S., Hansen E. G., Fichter K. (2021). University-linked programmes for sustainable entrepreneurship and regional development: how and with what impact?. *Small Business Economics*.

[21] Chang T. Y., Hong G., Paganelli C. (2021). Innovation of dental education during COVID-19 pandemic. *Journal of Dental Sciences*.

